The article "Lycium barbarum polysaccharide induced apoptosis and inhibited proliferation in infantile hemangioma endothelial cells via down-regulation of PI3K/AKT signaling pathway" was retracted in 2024. Reasons: duplicated images; concerns about the images.

# *Lycium barbarum* polysaccharide induced apoptosis and inhibited proliferation in infantile hemangioma endothelial cells via down-regulation of PI3K/AKT signaling pathway

**DOI:** 10.1042/BSR20191182

**Published:** 2019-08-19

**Authors:** Lin Lou, Guo Chen, Bing Zhong, Feng Liu

**Affiliations:** 1 Department of Oto-Rhino-Laryngology, West China Hospital, West China Medical School, Sichuan University China, No. 37 Guo Xue Alley, Chengdu City 610041, Sichuan Province, China; 2 Department of Otorhinolaryngology Head and Neck Surgery, The People’s Hospital of Jianyang City, No. 180, Hospital Road, Jianyang City 641400, Sichuan Province, China

**Keywords:** apoptosis, HemECs, Infantile hemangioma, Lycium barbarum polysaccharide, PI3K/AKT signal pathway

## Abstract

*Lycium barbarum* polysaccharide (LBP) has a variety of pharmacological and biological activities such as anti-inflammatory, antioxidation, anti-apoptosis, immune regulation and other pharmacological effects; however, the effect of LBP on infantile hemangioma (IH) was less reported. Primary human hemangioma endothelial cells (HemECs) were isolated from fresh surgical specimens of patients. HemECs was treated with LBP and the changes in proliferative and apoptotic signaling pathways were investigated by performing cell counting kit-8, cloning formation experiment, *in vitro* angiogenesis experiment, flow cytometry, Western blot, immunofluorescence, HE stain and real-time quantitative polymerase chain reaction. We found that LBP potently inhibited the proliferation of HemECs and achieved a low-micromolar IC_50_ (45 and 40 μg/ml, the half maximal inhibitory concentration) value and less angiogenesis, however, the IC_50_ had no effect on human umbilical vein endothelial cells (HUVECs) viability. LBP treatment induced apoptosis in HemECs, which was supported by positive Annexin-V-FITC staining, the activation of cleaved caspase-3 and Bcl-2-associated X protein (Bax) and the inhibition of B-cell lymphoma/leukemia-2 (Bcl-2). Moreover, the result demonstrated that LBP suppressed the expressions of proliferating cell nuclear antigen (PCNA), Ki67, vascular endothelial growth factor (VEGF), VEGFR2 and phosphoinositide 3-kinase (PI3K)/protein kinase B (Akt) signal pathway. PI3K-specific agonist (IGF-1) had promotive effects on HemECs proliferation, which was reversed by LBP. Our study suggests that the effectiveness of LBP in IHs may be associated with its potent anti-proliferative and apoptotic activities in HemECs. Thus, our findings may provide an effective medicine for IHs treatment.

## Introduction

Infantile hemangioma (IH) is the most frequent benign tumor in infants and young children, and the incidence of IH is approximately 3–10% [1]. Study found that women, Caucasians, low-weight premature infants, multiple births and elder infants are more susceptible to have the disease [2]. Potential complications of IH are, for example, permanent disfigurement, ulcers, scarring, bleeding, visual impairment, airway obstruction, congestive heart failure, in some cases, IH could even cause death [3]. Approximately 10% of all IH cases complete their own degradation within 1 year, while the remaining 90% IH cases take 3–10 years or longer to degrade [4]. Most of regressed tumors leave a mark that affects aesthetics or fibrous fat deposits [5]. Therefore, researchers tend to actively intervene in the early stage of IH to promote and accelerate the spontaneous regression process of the disease and reduce the invasion of vascular tumors on surrounding woven tissues [6–8].

*Lycium barbarum* polysaccharide (LBP) is a macromolecular substance with a variety of biological activities extracted from the traditional Chinese herb *Lycium barbarum*. LBP has functions of antitumor, antioxidation, anti-free radicals, sugar lipid-lowering and other pharmacological activities [9,10]. Previous study showed that LBP could bind to the polysaccharide receptors, which was present on the surface of dendritic cells (DCs) [11], and that activated DCs and their released active factors indirectly affect T cells to improve their activities, thus, T cells are transformed into killer T cells to increase the killing ability of T cells [12]. LBP can also directly act on tumor cells, and by directly destroying the membrane surface structure of cancer cells, tumor cells cannot perform normal life activities and the fluidity of tumor cell membranes was therefore reduced [13–15]. However, there are few researches conducted on the effects of LBP on IH endothelial cells (hemangioma endothelial cells (HemECs)).

Activation of phosphatidylinositol 3-kinase (PI3K)/AKT signaling pathway up-regulates the expressions of vascular endothelial growth factor (VEGF) and VEGF receptor 2 in neural progenitor cells and brain endothelial cells and promotes angiogenesis [16]. PI3K/AKT signaling pathway is involved in the regulation of various cellular functions such as proliferation, differentiation, apoptosis and glucose transport [17]. In recent years, PI3K has been found to be closely related to tumor angiogenesis and the degradation of extracellular matrix [18,19]. Activated AKT activates or inhibits its downstream target proteins, for example, Bad and Caspase 9, by acidification to regulate cell proliferation, differentiation, apoptosis and migration [20].

Focusing on cell apoptosis and PI3K/AKT signaling pathway, the present study aimed to investigate the molecular mechanism of LBP protection against HemECs. Our findings provide new insights into and theoretical basis for the development of natural drugs for the treatment of IH.

## Materials and methods

### Tissue samples and HemECs identification

IH tissues were obtained from fresh surgical specimens of three patients, the age of the three patients was less than 6 months. The diagnosis of IH of these patients was made based upon clinical examination and computed tomography with and without contrast in the West China Hospital, West China Medical School, Sichuan University China. The study was approved by the West China Hospital, West China Medical School, Sichuan University China Ethics Committee and the consents were signed by the parents of those three patients. The tumor tissues were cut into 2 × 2 mm pieces and placed in a digestive solution containing 0.2% collagenase A for digestion. Cells with positive expressions were used as the specific markers of factor VIII (anti-factor VIII, rabbit; 1:100; ab236284; Abcam), CD31 (anti-CD31, rabbit; 1:50; ab28364; Abcam) and CD34 (anti-CD34, rabbit; 1:100; ab81289; Abcam) hemangiomas were sorted by using flow cytometry. The positive cells were incubated with EGM-2V (Lonza, U.S.A.) containing 20% FBS (Gibco, Solarbio, Beijing), SingleQuot (Hefg, VEFG, hFGF-B, ascorbic acid, heparin and gentamicin/amphotericin) and PS at 37°C in 5% CO_2_.

### Cells culture

The HemECs were plated in RPMI 1640 supplemented with 10% heat-inactivated FBS, streptomycin (100 mg/ml, Solarbio, Beijing) and penicillin (100 U/ml, Solarbio, Beijing). Human umbilical vein endothelial cells (HUVECs) were purchased from MT Biological Technology Co. (http://www.mt-bio.com/en/index.aspx, Shanghai, China) and cultured in DMEM containing 10% FBS. Cell culture was conducted in an incubator at 37°C with 5% CO_2_.

### Reagent

LBP was purchased from QiYuan Pharmaceutical of Ningxia Hui Autonomous Region (purity ≥ 97% by HPLC, Yinchuan, China). IGF-1 was purchased from Sigma (121767, purity ≥ 98% by HPLC, Sigma–Aldrich, St. Louis, MO, U.S.A.).

### Immunohistochemistry

Cells in logarithmic growth phase were seeded in a six-well plate at a cell density (2 × 10^6^) of each well, fixed with 4% paraformaldehyde for 10 min, rinsed three times with PBS and then incubated with 0.1% Triton X-100 for 10 min. The cells were stained with primary antibodies (factor VIII, CD31 and CD34) and then washed and stained with secondary antibody. Cells were stained with Hematoxylin and Eosin (H&E) for histological analysis were observed by a Leica CTR6000 microscope.

### CCK-8 assay

The cells were seeded at 4 × 10^3^ cells/well in a 96-well plate (culture medium 100 μl/well), which was incubated overnight in an incubator. Ten microliters of CCK-8 (Beyotime Institute of Biotechnology, Beijing, China) was added into each well, and the plates were incubated for 2 h in an incubator. The absorbance at 450 nm was measured using a microplate reader (Tecan Infinite M200 Micro Plate Reader; LabX, Männedorf, Switzerland).

### Cloning formation assay

After HemECs were treated with LBP, 800 cells were inoculated into six-well plates, and each group was set up with three replicate wells. The cells were cultured in an incubator for 2 weeks in 5% CO_2_ at 37°C (the culture solution was changed every 2 days). The medium was aspirated, and 500 μl methanol solution was then added into each well to fix the cells for 15 min, the methanol was discarded and 1 ml Crystal Violet dye solution was added into each well to stain the cells for 20 min. The enzyme-linked spot image automatic analyzer was used to scan and photograph.

### Annexin V/PI staining

HemECs were transferred to a centrifugation tube and centrifuged at 1000×***g*** for 4 min at room temperature, and the supernatant was discarded and washed with physiological saline once. A total of 500 μl of 1× binding buffer was added to the pelleted cells according to the instructions of cell apoptosis detection kit (K201-100, BioVision, Milpitas, CA, U.S.A.). The cells were then incubated with 10 μl FITC-labeled Annexin V and 5 μl PI in the dark for 10 min at room temperature, and the results were immediately measured by flow cytometry. The collected cells were divided into four quadrants as follows: living cells (Annexin V^−^/PI^−^) were in the lower left quadrant, early apoptotic cells (Annexin V^+^/PI^−^) were in the lower right quadrant, the upper right quadrant contained late apoptotic cells (Annexin V^+^/PI^+^) and the upper left quadrant contained necrotic cells (Annexin V^−^/PI^+^).

### H&E staining

HemECs were treated with LBP (45 μg/ml) for 24 h, and then HemECs in logarithmic growth phase were harvested. The cells were digested with trypsin, and a single cell suspension at a density of 5 × 10^4^ cells/ml was prepared after digestion. The circular glass slices were placed in six-well plates, cell suspensions were added and then cultured in an incubator for 3 h in 5% CO_2_ at 37°C to make cells climbing pieces. Subsequently, the cells climbing pieces were removed and washed three times with PBS, fixed with 4% paraformaldehyde for 15 min, washed with PBS for three times, stained with Hematoxylin for 10 min and washed with PBS for three times. The cells climbing pieces were treated with xylene for 15 min, stained with Hematoxylin for 2 min, combined with 1% hydrochloric acid ethanol for 1–3 s, slightly washed for 1–2 s and stained by 0.5% Eosin solution for 2–3 min. The glass slides were placed into gradient concentrations of ethanol (80, 95 and 100%) for 2 min each for dehydration, transparentized with xylene I, II for 3 min and finally sealed with neutral gel.

### Tube experiment

Matrigel gel (Corning) was dissolved at low temperature, and 10 μl Matrigel was added to the well. The 96-well plate coated with Matrigel gel was placed at 37°C and incubated in 5% CO_2_. After 30 min, 100 μl of cell suspension with at a cell concentration of 5 × 10^4^ was added to each well and photographs were taken 4 h later.

### ELISA

The VEGF (P58294, RayBiotech, Norcross, GA, United States) and VEGFR2 (P35968, RayBiotech) in the cell lysates were determined by ELISA kit. The assays were conducted in duplicate according to the manufacturer’s protocols.

### Western blot analysis

HemECs were washed twice with pre-cooled saline, and the liquid in each bottle was aspirated as much as possible, and 500 μl of pre-cooled lysis buffer (RIPA, Santa Cruz, CA, United States) was then added. The mixture was allowed to stand for 40 min in an ice bath and then centrifuged at 12000×***g*** at 4°C for 20 min to collect total protein. The supernatant protein concentration was determined by BCA assay (Biyuntian). Thirty micrograms of protein was subjected to 10% SDS/polyacrylamide gel electrophoresis and transferred to a PVDF membrane (Nanjing Institute of Bioengineering, China), which was blocked with 5% skimmed milk powder for 2 h at room temperature, and anti-B-cell lymphoma/leukemia-2 (Bcl-2)-associated X protein (Bax) (21 kDa; rabbit; 1:1000; ab32503; abcam), anti-Bcl-2 (26 kDa; rabbit; 1:1000; ab32124; abcam), anti-C caspase-3 (17 kDa; rabbit; 1:1000; ab2302; abcam), anti-Ki-67 (359 kDa; rabbit; 1:1000; ab92742; abcam), anti-proliferating cell nuclear antigen (PCNA) (39 kDa; rabbit; 1:1000; ab18197; abcam), anti-p-PI3K (85 kDa; rabbit; 1:1000; #4228; CST), anti-PI3K (85 kDa; rabbit; 1:1000; #4292; CST), anti-p-protein kinase B (Akt) (60 kDa; rabbit; 1:1000; #9271; CST), anti-Akt (60 kDa; rabbit; 1:1000; #9272; CST) and anti-GAPDH (36 kDa; mouse; 1:1000; ab8245; abcam) were added to corresponding target strips and incubated overnight at 4°C. After washing the cells by TBS, horseradish peroxidase-labeled goat anti-rabbit or mouse IgG (1:5000, sc-516102/sc-2357; Santa Cruz Biotechnology, Inc. Dallas, TX, U.S.A.) was incubated with the target strips at 37°C for 2 h. The target strips were developed by ECL kit (Biyuntian Biotechnology Co., Ltd.), and strip gray value was calculated by ImageJ.

### Real-time quantitative PCR

One milliliter of TRIzol lysate was added to lyse the HemECs for collecting total RNA. Supernatant was collected, 200 μl of chloroform was added to the supernatant and held for 5 min at room temperature and centrifuged together at 12000×***g*** for 15 min at 4°C. The upper layer of liquid was drawn and transferred to a new centrifugation tube, 500 μl of isopropanol was added and held at room temperature for 10 min and then centrifuged at 12000×***g*** for 10 min at 4°C. The supernatant was discarded and the precipitate was washed with 1 ml of 75% ethanol (anhydrous ethanol and DEPC-treated water) and centrifuged at 7500×***g*** for 5 min at 4°C. Next, 25 μl DEPC water was added and total RNA concentration was measured by Nandrop (A260/A280 was between 1.8 and 2.0). The total RNA was extracted from TRIzol for reverse transcription reaction at 42°C for 10 min and at 95°C for 15 min and stored at 4°C. SYBR Green PCR Master Mix (Roche, Basel, Switzerland) was used to conduct qPCR experiment using opticon RT-PCR detection system (ABI 7500, Life Technology, U.S.A.), and the PCR cycles were as follows: pretreatment at 95°C for 10 min, followed by 40 cycles at 94°C for 15 s, 60°C for 1 min, finally at 60°C for 1 min and preserved at 4°C. The gene copy number of each sample was expressed by *C*_t_ value, and the relative expression of gene was analyzed by the 2^−ΔΔ*C*^_q_ method [21]. The primers are listed in Table 1.

**Table 1:** Primers for RT-qPCR

Genes	Forward (5′–3′)	Reverse (5′–3′)
*Bax*	TTCTGACGGCAACTTCAACT	CAGCCCATGATGGTTCTGAT
*Bcl-2*	ATGTGTGTGGAGAGCGTCAA	GAGACAGCCAGGAGAAATCAA
*PCNA*	CCTGCTGGGATATTAGCTCCA	CAGCGGTAGGTGTCGAAGC
*Ki67*	GCCTGCTCGACCCTACAGA	GCTTGTCAACTGCGGTTGC
*GAPDH*	CACCCACTCCTCCACCTTTG	CCACCACCCTGTTGCTGTAG

### Statistical analysis

The results were shown as the mean ± SD. Statistical significance was determined by analysis of variance (ANOVA) between groups, followed by Dunnett’s *t* test using GraphPad Prism (GraphPad Software Inc., La Jolla, CA, U.S.A.). *P<0.05* was considered as statistically significant.

## Results

### HemECs viability was inhibited by LBP in a dose-dependent manner

To verify that the cells isolated from IH tissue were HemECs, the expressions of factor VIII, CD31 and CD34 in the cells were examined by immunofluorescent staining. We found that all cells expressed three molecules and had high intensities (Figure 1A). As these three cell-surface molecules were used as biomarkers for the identification of endothelial cells, and data suggested that most cells isolated from IH tissues were HemECs and could be used in further investigation. To examine the inhibitory effect of LBP on the proliferation of HemECs and HUVECs, the cells were treated with LBP (0–500 μg/ml) for 24 and 48 h, and cell viability was examined by CCK-8 assay. The results showed that LBP suppressed cell viability in HemECs and HUVECs at 24 h (Figure 1B) and 48 h (Figure 1C). However, when half maximal inhibitory concentration (IC_50_) values were 45 and 40 μg/ml at 24 and 48 h, the activity of LBP was much stronger in HemECs, compared with that in HUVECs. Thus, 45 μg/ml LBP was used in later experiments.

**Figure 1:** HemECs viability was inhibited by LBP in a dose-dependent manner (**A**) The expressions of factor VIII, anti-CD31 and anti-CD34 were determined by immunofluorescence analysis (magnification ×400). (**B**) HemECs and HUVECs were treated with LBP at concentrations of 0, 20, 50, 100, 200 and 500 μg/ml for 24 h. Cell viability was determined using the CCK-8 assay. (**C**) HemECs and HUVECs were treated with LBP at concentrations of 0, 20, 50, 100, 200 and 500 μg/ml for 48 h, and cell viability was determined using CCK-8 assay. **P<0.01 vs 0 μg/ml.

### HemECs proliferation was inhibited and apoptosis was induced by LBP in a dose-dependent manner

We further performed cloning formation experiment and flow cytometry to visualize the effects of LBP on the HemECs proliferation and apoptosis, we noted that LPB treatment inhibited cell proliferation in a dose-dependent manner (Figure 2A,B). Treating cells with LBP using Annexin-V-FITC and PI staining led to a significantly increased apoptosis of HemEC, compared with the control (Figure 2C,D).

**Figure 2:** HemECs proliferation was inhibited and apoptosis was induced by LBP in a dose-dependent manner (**A**) HemECs were treated with LBP at concentrations of 0, 20, 50, 100, 200 and 500 μg/ml. (**B**) Cell proliferation was determined and quantified by cloning formation assay. (**C**) HemECs were treated with LBP at concentrations of 0, 20, 50, 100, 200 and 500 μg/ml, and cell apoptosis was determined and quantified (**D**) using flow cytometry. *P<0.05, **P<0.01 vs 0 μg/ml.

### HemECs growth and angiogenesis were inhibited by LBP

To further investigate the potential biological effects of LBP on HemECs, the effects of LBP on HemECs growth was investigated and tube formation and the expression levels of PCNA, Ki-67, Bcl-2, Bax and c caspase-3 were determined. We observed that HemECs grow slowly and sparsely distributed when exposed to LBP, and that the colony growth was not as obvious as in the control group (Figure 3A). In HemECs, the mRNA levels of PCNA, Ki-67 and Bcl-2 were up-regulated, while the mRNA level of Bax was down-regulated. However, those phenomena were reversed by LBP (Figure 3B). The protein levels of PCNA, Ki-67 and Bcl-2 were lower but the levels of Bax and c caspase-3 were higher in HemECs+LBP group than those in HemECs group (Figure 3C,D). The data from tube formation showed that angiogenesis in HemECs was inhibited by LBP (Figure 3E,F).

**Figure 3:** HemECs growth and angiogenesis were inhibited by LBP (**A**) HemECs were treated with LBP at concentrations of 45 μg/ml (IC_50_) for 24 h, and the morphology was observed using H&E staining. (**B**) The mRNA levels of PCNA, Ki-67, Bcl-2 and Bax were analyzed by RT-qPCR. The protein levels of PCNA, Ki-67, Bcl-2, Bax and C caspase-3 were determined (**C**) and quantified (**D**) by Western blot. HemECs and HUVECs angiogenesis was determined (**E**) and quantified (**F**) by tube experiment. **P<0.01 vs HUVECs, ^##^*P<*0.01 vs HemECs.

### LBP affected VEGF, VEGFR2, p-PI3K and p-Akt protein expression in HemECs

We found that LBP caused a decrease in angiogenesis in HemECs. The levels of VEGF and VEGFR2 were determined by ELISA, and the data showed that the increase in VEGF (Figure 4A) and VEGFR2 (Figure 4B) in HemECs were prevented by LBP. Furthermore, we examined whether PI3K/Akt signal pathway was involved in the protection of LBP to HemECs, and found that the protein expressions of p-PI3K and p-Akt were greatly induced in HemECs, and that LBP significantly suppressed the protein expressions of p-PI3K and p-Akt in HemECs (Figure 4C–F).

**Figure 4:** LBP affects the protein expressions of VEGF, VEGFR2, p-PI3K and p-Akt in HemECs The expressions of (**A**) VEGF and (**B**) VEGFR2 were determined using ELISA. (**C**) The protein levels of (p)-PI3K and (p)-Akt were determined by Western blot. The relative levels of proteins described in (**D**) were counted by GAPDH as normalization. The relative levels of p-PI3K described in (**E**) were counted by PI3K as normalization. The relative levels of p-Akt described in (**F**) were counted by Akt as normalization. **P<0.01 vs HUVECs, ^##^*P<*0.01 vs HemECs.

### LBP partially reversed the proliferative effects of IGF-1 in HemECs

In order to confirm the role of PI3K/Akt signal pathway in HemECs progression, after cells were treated with or without LBP for 24 h, IGF-1 was used to treat HemECs. The functional experiments were analyzed by cloning formation experiment, flow cytometry, Western blot, tube formation and ELISA. When the IGF-1 was added to cell culture medium, the inhibition of LBP on proliferation of HemECs was reversed (Figure 5A,B). The data from flow cytometry showed that IGF-1 had no effect on HemECs apoptosis, LBP significantly promoted HemECs apoptosis, and the promotion of LBP on apoptosis of HemECs was reversed by IGF-1 (Figure 5C,D). The protein levels of PCNA, Ki-67 and Bcl-2 were lower but the protein levels of Bax and c caspase-3 were higher in IGF-1+LBP group than those in IGF-1 group (Figure 5E,F). The mRNA levels of PCNA, Ki-67 and Bcl-2 were up-regulated, while the mRNA level of Bax was down-regulated by IGF-1, however, those phenomena were reversed by LBP (Figure 5G). The data from tube formation showed that HemECs angiogenesis was promoted by IGF-1 but reversed by LBP (Figure 5H,I). ELISA data demonstrated that the increase in VEGF caused by IGF-1 (Figure 5J) and VEGFR2 (Figure 5K) in HemECs were inhibited by LBP.

**Figure 5:** LBP partially reversed the proliferative effects of IGF-1 in HemECs HemECs were treated with LBP or/and IGF-1, and cell proliferation was determined (**A**) and quantified (**B**) by cloning formation assay. Cell apoptosis was determined (**C**) and quantified (**D**) using flow cytometry. The protein levels of PCNA, Ki-67, Bcl-2, Bax and C caspase-3 were determined (**E**) and quantified (**F**) by Western blot. (**G**) The mRNA levels of PCNA, Ki-67, Bcl-2 and Bax were determined by RT-qPCR. HemECs and HUVECs angiogenesis were determined (**H**) and quantified (**I**) by tube experiment. The expressions of (**J**) VEGF and (**K**) VEGFR2 were determined by ELISA. **P<0.01 vs Control, ^##^*P<*0.01 vs IGF-1, ^∧∧^*P<*0.01 vs LBP.

## Discussion

IH is one of the most common vascular tumors among infants, and the pathogenesis of IH is complex. Various antenatal related factors were found to be risk factors of IH in previous studies, such as placenta previa, progesterone use and preeclampsia [2,22]. Clinical manifestations of IH may vary, but a few lesions cause damage to important functions (such as respiratory or visual impairment), permanent scarring or disfigurement [23]. Thus, effective treatment is necessary. The pathological feature of IH is that endothelial cells proliferate rapidly at the initial stage and then enter the slow degradation stage [24]. The abnormal structure and function of endothelial cells may cause diseases such as thrombosis, atherosclerosis and vasculitis, thus, it is important to isolate and culture endothelial cells *in vitro* [25]. HUVECs are involved in many fields of research and is widely used in studying vascular diseases [26]. HUVECs are used for the investigation of vascular endothelial function [27], blood supply of flaps [28] and tissue blood supply after radiotherapy [29]. In this study, HemEC was isolated and cultured in order to establish a comparative study of endothelial vasospasm in IH. The biological time difference between vascular endothelial cells of IH and vascular endothelial cells of normal tissues was compared. In 1982, Mulliken et al. [30] found the isolation of vascular endothelial cells from hemangiomas and vascular malformations and reported the characteristics of tubes *in vitro*. Similarly, we successfully isolated positive hepatoma endothelial cells in CD31, CD34 and factor VIII for subsequent experiments.

LBP has a variety of biological characteristics including antioxidation, anti-apoptosis, immune regulation and other pharmacological effects [31,32]. It has been reported that LBP has anticancer properties. For example, LBP induces apoptosis and inhibits proliferation of human hepatoma QGY7703 cells [33]; LBP inhibits the proliferation of HeLa cells by inducing apoptosis through the mitochondrial pathway [34]. Zhang et al. [14] reported that LBP has an inhibitory effect on the growth of human hepatoma SMMC-7721 cells. These data indicated that LBP had a potential anti-proliferative capacity. It has been shown that apoptotic resistance was an important characteristic of proliferative IH endothelial cells [35]. Our data showed that LBP treatment led to cells proliferation inhibition, Annexin-V-positive staining and changes in related proteins in HemECs, in addition, LBP also exhibited a degree of selectivity in targeting HemECs rather than HUVECs. We speculated that the selectivity could be attributed to the abnormal cellular structure and the rapid dividing nature of HemEC. Our findings indicated that LBP could be used to treat patients with IH. However, the underlying mechanism should be specifically determined. In addition, studies have reported that LBP has an anti-apoptotic effect. LBP not only prevents cisplatin-induced MLTC-1 cell apoptosis and autophagy by regulating endoplasmic reticulum stress pathway [36], but also protects human lens epithelial cells from H_2_O_2_-induced apoptosis [37]. Jing and Jia [38] reported that LBP inhibits palmitate-induced apoptosis in MC3T3–E1 cells by decreasing the activation of ERS–mediated apoptosis pathway. Whether LBP acts as an anti-apoptotic or pro-apoptotic agent may be determined by different cells.

Upon the activation of VEGF and VEGFR-2 in HemECs, PI3K/Akt signaling pathways trigger multiple downstream signals that promote angiogenesis [39]. Medici and Olsen [40] found that HemECs constitutively activate PI3K/Akt aix. Propranolol induces the regression of hemangioma cells by down-regulating PI3K/Akt pathway [41]. Moreover, LBP attenuates diabetic testicular dysfunction through the inhibition of PI3K/Akt pathway [42,43]. We showed that LBP also effectively suppressed the phosphorylation of PI3K and Akt in HemECs, and that the promotion of IGF-1 (Akt-specific activatior) in HemECs was reversed by LBP. These findings suggested that the inhibitory effect of LBP on the proliferation of HemECs may be correlated to PI3K/Akt pathway. Additional investigations in cellular levels are required to determine detailed molecular targets that mediate anti-apoptotic effects of LBP.

To conclude, our study demonstrated that LBP showed potent anti-proliferative and apoptosis activities in HemECs by the inhibition of PI3K/Akt signal pathway. Our findings provide a rational basis to the clinical application of LBP in the treatment of IHs and also provided insight into the understanding of the cellular and molecular mechanisms of LBP in the treatment of IH.

## Abbreviations

Akt: protein kinase B
Bax: Bcl-2-associated X protein
Bcl-2: B-cell lymphoma/leukemia-2
CCK-8: cell counting kit-8
DC: dendritic cell
DEPC: diethylpyrocarbonate
ERS: endoplasmic reticulum stress
GAPDH: glyceraldehyde-3-phosphate dehydrogenase
HE: hematoxylin and eosin
HemEC: hemangioma endothelial cell
HUVEC: human umbilical vein endothelial cell
IGF-1: insulin-like growth factors-1
IH: infantile hemangioma
LBP: *Lycium barbarum* polysaccharide
MLTC-1: Murine leydig tumor cell line-1
PCNA: proliferating cell nuclear antigen
PI3K: phosphoinositide 3-kinase
PI: propidium iodide
qPCR: quantitative polymerase chain reaction
VEGF: vascular endothelial growth factor
VEGFR2: vascular endothelial growth factor receptor 2
